RETRACTED

# miR-211-5p Alleviates the Myocardial Ischemia Injury Induced by Ischemic Reperfusion Treatment via Targeting FBXW7

**DOI:** 10.1155/2022/5423929

**Published:** 2022-06-03

**Authors:** Yonghui Liu, Jiatian Meng, Hongqin Di, Liheng Zheng, Zili Meng

**Affiliations:** ^1^Department of Cardiovascular Surgery, Hebei Chest Hospital, Hebei Lung Cancer Research Center, Shijiazhuang, 050041 Hebei, China; ^2^Department of Radiology, Hebei Chest Hospital, Hebei Lung Cancer Research Center, Shijiazhuang, 050041 Hebei, China; ^3^Molecular Biology Laboratory, Hebei Chest Hospital, Hebei Lung Cancer Research Center, Shijiazhuang, 050041 Hebei, China; ^4^Department of Laboratory, Hebei Chest Hospital, Hebei Lung Cancer Research Center, Shijiazhuang, 050041 Hebei, China

## Abstract

Cardiovascular diseases, a class of the most common diseases, seriously threaten human health, which is a direct inducement of death in most countries. The restoration of blood supply is an impactful intervention way for cardiovascular disease treatments while the injury induced by oxygen-glucose deprivation and ischemic reperfusion (I/R) may further impact the tissues of the patients. Myocardial reperfusion is a precondition for saving ischemic myocardial tissues in acute myocardial infarction while the injury induced by immediate reperfusion takes a great challenge for cardiovascular disease treatment. Howbeit, the reperfusion of coronary blood could aggravate the injury triggered by ischemia. At present, several studies have focused on the etiopathogenesis and therapeutic strategies of ischemia-reperfusion injury of the myocardium. The report has verified that miR-211-5p was elevated in the pathological specimens, while the influence of miR-211-5p in I/R-mediated injury of myocardial cells remains unclear. This research is aimed at illustrating the role of miR-211-5p in the progression of I/R injury of myocardial cells, and qRT-PCR, western blot, CCK-8, and TUNEL assay were used to investigate the functions of miR-211-5p on I/R-mediated injury of myocardial cells. The result mirrored that miR-211-5p was distinctly reduced in the I/R-induced AC16, and reduced miR-211-5p could evidently improve the viability of I/R-induced AC16. miR-211-5p could directly target FBXW7, and FBXW7 upregulation could reverse the improvement of AC16 in viability and apoptosis level after suffering I/R. Moreover, it was also proved that miR-211-5p can mediate the activation of Wnt/*β*-catenin via attenuating FBXW7. Consequently, this investigation identified miR-211-5p as a positive role to attenuate the injury of myocardial cells when suffering I/R treatment.

## 1. Introduction

Cardiovascular diseases, a class of the most common diseases, seriously threaten human health, which is a direct inducement of death in most countries [1, 2]. At present, surgery and drug interventions are major strategies for cardiovascular disease, and the restoration of blood supply effectively reduced the damage and the infarct induced by ischemic reperfusion (I/R), thus minimizing the rate of mortality [3, 4]. However, the research has shown that immediate blood supply may cause extra cardiovascular trauma in patients, which can trigger some harmful events such as myocyte apoptosis and even cardiac arrest [5]. Consequently, it remains valuable to delve the corresponding theory underlying this pathema and to examine the practical values of conceivable strategies that alleviate myocardial I/R injury.

RETRACTED

In recent ten years, the roles of noncoding RNA in the progression of diseases have been found, and the regulation of those factors has also been confirmed as effective strategies for treatments of multiple diseases [6]. MicroRNAs (miRNAs) can negatively influence gene abundance by mediating the deterioration of mRNAs, effectively inhibiting protein translation [7, 8]. Several researches have evidenced that miRNA dysfunction is associated with the formation and development of cardiovascular disease, and they are also involved in the progression of the apoptosis and inflammation of myocardial cells induced by ischemic reperfusion [8, 9]. A previous report has evidenced the reduced miR-211-5p in PC12 cells after I/R treatment [10]. Nevertheless, the role of miR-211-5p in the development of ischemic reperfusion injury remains unclear. Analogously, the investigation also evidenced that miR-211-5p was dramatically reduced in IR-induced human kidney cells. Moreover, miR-211-5p has also been recognized as a protector to keep neonates from heart injury induced by ischemia, suggesting that decreased miR-211-5p may be related to the jury of cardiomyocytes.

This research arranged to investigate the connection of miR-211-5p and the ischemic reperfusion injury of myocardial cells and mirrored the corresponding characteristics of miR-211-5p in the ischemic reperfusion injury of myocardial cells. Moreover, this research determined that miR-211-5p could induce the activation of Wnt pathway while this phenomenon could be abolished by FBXW7 upregulation. It has been found that FBXW7 serves as an inhibitor to suppress the activation of Wnt pathway in lung cancer [11]. Hence, this study sustains that attenuated miR-211-5p can promote the injury and apoptosis of myocardial cells suffering I/R via regulating FBXW7 mediated the inactivation of Wnt pathway [12].

## 2. Material and Methods

### 2.1. Cells and Cell Models

AC16, the human cardiomyocyte cell line (Manassas, VA, USA), was selected for model establishment. DMEM (Gibco, NY, USA) was selected as medium. Besides, 10% fetal bovine serum (FBS) was applied to maintain cell growth. Finally, the cells were cultured in a condition with 5% CO_2_ and 37°C. AC16 cells were treated with 94% N_2_, 5% CO_2_, and 1% O_2_ for 6, 12, and 24 h to establish the ischemic cell models.

RETRACTED

### 2.2. Cell Transfection

Six-well plates was applied to cell culture, and the miR-211-5p mimics pcDNA-FBXW7 and the related negative controls (NCs) were transfected added into the related well (cellular confluence: 70%). Briefly, the transfectants and Lipofectamine 2000 were thinned with 250 *μ*l medium, respectively. Subsequently, the thinned transfectants were mixed with Lipofectamine 2000 diluent (1 : 1). Immediately, the mixtures stood at 25°Cfor 20 min. Immediately, 500 *μ*l of the incubated transfectants was added in related wells. Finally, the cells were cultured for the subsequent experiments.

### 2.3. qRT-PCR

TRIzol (Sobao Biological Technology Co., Ltd., Shanghai, China) was selected for RNA extraction, and the RNAs were quantified with spectrophotometry. Subsequently, cDNA reverse transcription was executed with the commercial kit (MBL Beijing Biotech Co., Ltd., China). Besides, the primers were provided by RiboBio (Guangzhou, China). After that, the PCR reaction systems were prepared referred to the instruction of the kit (Sigma-Aldrich, Missouri, USA). Besides, the parameters of reactions are as follows: denaturation (95°C, 3 min), amplification (95°C for 12 s and at 53°C for 40 s), and final 70°C for 30 s. Ultimately, the 2^−(*ΔΔ*Ct)^ method was applied to quantification of miRNAs. The information of the primers is displayed in Table 1.

### 2.4. Western Blot

RIPA solution was applied to protein extraction at 4°C. The commercial BCA kit (Borf Biotechnology Co., Ltd., Wuhan, China) was applied to the protein quantification. After that, the thermal denaturation of the proteins was executed for 5 min. Protein isolation was performed by SDS-PAGE gels, and then, the wet transfer method was applied to transmembrane. Immediately, the membranes blocking were executed with 5% milk (no fat) for 1 h. After that, the membrane incubation was executed with the first and second antibodies in turn. Finally, a chemiluminescence detection system was applied to quantify the abundances of targets. Antibody information is as follows: anti-FBXW7 (1 : 1000, ab2533451, ThermoFisher, Massachusetts, USA), anti-Wnt (1 : 1000, ab11154198, ThermoFisher, Massachusetts, USA), anti-*β*-catenin (1 : 1000, ab2533039, ThermoFisher, Massachusetts, USA), and cleaved Caspase-3 (1 : 1000, ab325431, ThermoFisher, Massachusetts, USA).

RETRACTED

### 2.5. Dual-Luciferase Reporter Assay

The mutant 3′-UTR sequences of FBXW7 were designed according to the prediction of the Targetscan database. Subsequently, the mutant types and related wild types were, respectively, linked with the pmirGLO vectors (Yanjiang Bio Co., Ltd., China) and named as FBXW7-mut and FBXW7-wt, respectively. Subsequently, FBXW7-mut or FBXW7-wt were, respectively, cotransfected with miR-211-5p mimics or the related NCs into the cells. Thereafter, the cells were incubated for 48 h. Ultimately, the luciferase activity of the cells was quantified.

### 2.6. TUNEL Assay

The 10% neutral formalin buffer was applied to cell fixation (25°C, 30 min), and then, the mixture of methanol and 0.3% H_2_O_2_ was applied to inactivate endogenous peroxidase. The cells were treated with permeabilizing solution (0.1% sodium citrate and 0.1% Triton X-100) at 4°C for 2 min. After that, the cells were treated with the reagent of terminal transferase-mediated biotin dUTP nick end labeling (TUNEL) at 37°C for 1 h. Finally, the Leica fluorescence microscope (Wetzlar, Germany) was applied to investigate cellular apoptosis.

### 2.7. CCK-8 Assay

CCK-8 Kit was provided by Amyjet (Wuhan, China). Firstly, the cells were cultured in 96-well plates (5 × 10^4^/well). Secondly, after transfection and I/R intervention, the cells were treated with CCK-8 reagent (10 *μ*L/well). Immediately, the cells were incubated for 4 h. Ultimately, cellular absorbance measurement (450 nm) was executed by a microplate reader (Molecular Devices, Shanghai, China).

### 2.8. Statistical Analysis

All experiments were repeated 3 times. Moreover, SPSS 20.0 and Graphpad Prism 8.0 were applied to data analysis and visualization, respectively. Besides, the difference of the data was tested with Chi-squared test or ANOVA with Tukey's post hoc-test. Moreover, *P* < 0.05 represented the difference was significant.

## 3. Results

### 3.1. Reduced miR-211-5p Was Detected in Patients' Serums

The abundance of miR-211-5p in patients' serums was quantified to reveal the relationship of miR-211-5p disorder and ischemic cardiomyopathy. The results mirrored that miR-211-5p was distinctly downregulated in patients' serums (Figure 1(a), *P* < 0.01). Then, AC16 cell models were established with I/R treatment. The results evidenced that the abundance of miR-211-5p was extremely reduced in I/R-treated cells (Figure 1(b), *P* < 0.01).

### 3.2. Reduced miR-211-5p Influenced the Phenotype of the Cells when Suffered I/R Treatment

To delve the miR-211-5p's functions in the development of myocardial inflammation, the miR-211-5p mimics were upregulated in I/R-induced cells, and the phenotype changing of I/R-treated cells was monitored. The CCK-8 reflected that miR-211-5p remarkably improved the viability of the I/R-treated cells. Besides, the TUNEL assay proved that miR-211-5p distinctly increased the apoptosis of I/R-treated cells (Figure 2, *P* < 0.01).

RETRACTED

### 3.3. miR-211-5p Was an Upregulator of FBXW7

The targets of miR-211-5p were screened through Targetscan. According to Targetscan, FBXW7 was screened as a target of miR-211-5p. Moreover, the luciferase assay was further applied to evidence the connection of miR-193-5p and FBXW7 (Figure 3(a), *P* < 0.01). Besides, the evidence proved that miR-211-5p could effectively affect the 3′-UTR of FBXW7. Besides, the decreased mRNA level of FBXW7 was also detected in I/R-treated cells (Figure 3(b), *P* < 0.01).

### 3.4. FBXW7 Abolished the Influences of miR-211-5p in the I/R-Treated Cells

Although the FBXW7 was proved as a target of miR-211-5p, whether FBXW7 was a pivotal downstream node of miR-211-5p in I/R-induced cells remains unknown. The miR-211-5p and FBXW7 were artificially upregulated in AC16 cells before I/R treatment, and the changes in cellular viability were monitored. Besides, the CCK-8 assay mirrored that reduced FBXW7 extremely inhibited the viability abolished the influence of reduced miR-211-5p on the I/R-treated cells (Figure 4(a), *P* < 0.01). Moreover, the TUNEL assay mirrored that the apoptosis of the cells contransfected with FBXW7 and miR-211-5p mimics was remarkably increased (Figure 4(b), *P* < 0.01).

### 3.5. miR-211-5p Was Involved in Wnt Pathway

For illustrating the related characters of miR-211-5p in the deterioration of myocardial ischemia injury, the abundance of the proteins in Wnt/*β*-catenin pathway was quantified. The results evidenced that reduced miR-211-5p remarkably attenuated the abundances of Wnt and *β*-catenin in AC16 cells, which could be abolished by FBXW7 downregulation (Figure 5, *P* < 0.01). Consequently, it suggested that attenuated miR-211-5p influenced the progression of myocardial ischemia injury via targeting FBXW7 mediated the inactivation of Wnt/*β*-catenin pathway.

## 4. Discussion

Myocardial reperfusion is a precondition for saving ischemic myocardial tissues in acute myocardial infarction while the injury induced by immediate reperfusion takes a great challenge for cardiovascular disease treatment [4, 13]. Howbeit, the reperfusion of coronary blood could aggravate the injury triggered by ischemia [14]. At present, several studies have focused on the etiopathogenesis and therapeutic strategies of ischemia-reperfusion injury of myocardium [2]. MicroRNAs (miRNAs) can negatively influence gene abundance via mediating the deterioration of mRNAs, effectively inhibiting protein translation. Several researches have evidenced that miRNA dysfunction is associated with the formation and development of cardiovascular disease, and they are also involved in the progression of the apoptosis and inflammation of myocardial cells induced by ischemic reperfusion. A previous report has evidenced the reduced miR-211-5p in PC12 cells after I/R treatment [10]. Nevertheless, the role of miR-211-5p in the development of ischemic reperfusion injury remains unclear. The study confirmed the connection between miR-211-5p and the injury in myocardial cells induced by ischemic reperfusion, revealed the target of miR-211-5p, and illustrated the related mechanism of miR-211-5p in the development of the ischemic reperfusion of myocardial cells.

RETRACTED

Several reports have indicated that the profiling of the miRNAs in myocardial cells exists visible difference before and after ischemic reperfusion [8]. Shan et al. have proved that the abundance of miR-93 in the myocardial cells induced by I/R treatment was extremely elevated, and miR-93 inhibition could effectively alleviate the injury on myocardial cells induced by oxidative stress and restrain the cellular apoptosis [15]. Analogously, the investigation also evidenced that miR-211-5p was dramatically reduced in IR-induced human kidney cells [16]. Moreover, miR-211-5p has also been recognized as a protector to keep neonates from heart injury induced by ischemia, suggesting that decreased miR-211-5p may be related to the jury of cardiomyocytes [17]. Thus, this report suggests that miR-211-5p can attenuate I/R-induced myocardial injury by targeting the downstream factors. The present evidences in this research reflected that miR-211-5p was an upregulation of FBXW7, and reduced FBXW7 was also observed in the myocardial cell induced by I/R treatment. This study also found that the changes induced by miR-211-5p in the phenotype of I/R-induced HBMECs could be abolished by elevated FBXW7. Besides, Tan et al. have observed that FBXW7 upregulation is related to the aberrant apoptosis of intestinal epithelial cells induced by I/R treatment, and reduced FBXW7 could effectively suppress the abundance of Caspase-3 and Caspase-9 in the IR-induced cells [18]. Therefore, this research sustains that miR-211-5p could attenuate the angiogenesis of HBMECs by reducing FBXW7. In this investigation, it was proved that the abundance of miR-211-5p in myocardial cells was extremely decreased after suffering I/R treatment. Moreover, it was also proved that increased miR-211-5p could significantly attenuate the apoptosis level and improve the viability of I/R-induced AC16 cells, which confirmed that miR-211-5p dysfunction plays a pivotal role in myocardial ischemia injury.

miRNA dysfunction has been proved as key reasons of development of many diseases, and increasing evidences have suggested the regulation of key proteins via impeding the transcription of the mRNAs [19]. Multifactorial regulation has also been proved as an important ability of the miRNA [20]. Besides, the function of miR-211-5p in protecting the brain tissues from I/R injury has been reported by a recent study. Interestingly, the recent report has evidenced the dramatically reduced miR-211-5p in the brains of I/R rat models, and elevated miR-211-5p can availably alleviate the focal cerebral injuries of the rats induced by I/R treatment via targeting COX2 [21].

RETRACTED

Several studies have indicated that miRNAs mediated progressions of diseases are related to the changes in activities of multiple pathways [22, 23]. Huang et al. have confirmed that miR-374a-mediated MAPK6 pathway inhibition could effectively protect mouse models away from injury of I/R treatment and reduce the apoptosis of myocardial cells [24]. In this investigation, reduced miR-211-5p was identified to inactivate Wnt pathway. Various researches have confirmed that the inactivation of Wnt pathway plays a key role in the injury and apoptosis process of the myocardial cells. The dysfunction of Wnt pathway has been also evidenced as a key reason of myocardial injury, and the study has found that miR-21/PDCD4 mediated the activation of Wnt pathway could effectively protect myocardial cells away from the damage and apoptosis induced by I/R treatment [25]. Moreover, this research determined that miR-211-5p could induce the activation of Wnt pathway while this phenomenon could be abolished by FBXW7 upregulation. It has been found that FBXW7 serves as an inhibitor to suppress the activation of Wnt pathway in lung cancer [11]. Hence, this study sustains that attenuated miR-211-5p can promote the injury and apoptosis of myocardial cells suffering I/R via regulating FBXW7 mediated the inactivation of Wnt pathway [12].

## 5. Conclusion

This study illustrated the role of miR-211-5p in myocardial ischemia injury triggered by I/R treatment and illustrated the related characters of miR-211-5p in protecting myocardial cells from I/R injury. It is suggested that miR-211-5p can attenuate the myocardial ischemia injury induced by ischemic reperfusion treatment via targeting FBXW7. However, this study still has limitations. The dysfunction of Wnt pathway has been also evidenced as a key reason of myocardial injury, but the mechanism of how it causes cardiomyocyte damage requires further studies to verify.

RETRACTED

## Figures and Tables

**Figure 1:** miR-211-5p was significantly reduced in I/R-induced AC16. (a) The relative abundance of miR-211-5p in the patients' serums. (b) The relative abundance of miR-211-5p was quantified by qRT-PCR (^∗∗^*P* < 0.01).

**Figure 2:** miR-211-5p attenuated the apoptosis of I/R-treated AC16. (a) The CCK-8 assay was applied to reveal the influence of miR-211-5p on the viability of I/R-induced AC16. (b) The influence of reduced miR-211-5p on the apoptosis of I/R-induced AC16 was analyzed by TUNEL (^∗∗^*P* < 0.01).

**Figure 3:** miR-211-5p acted as an upregulator of FBXW7, and FBXW7 was extremely elevated in I/R-induced AC16 cells. (a) The interaction of miR-211-5p and FBXW7 was verified by luciferase assay. (b) The quantification of FBXW7 by qRT-PCR (^∗∗^*P* < 0.01).

**Figure 4:** FBXW7 upregulation reversed the influence of reduced miR-211-5p in I/R-induced AC16 cells. (a) The viability of I/R-induced AC16 cells. (b) The apoptosis of I/R-induced AC16 (^∗∗^*P* < 0.01).

**Figure 5:** Reduced miR-211-5p induced the activation of Wnt pathway through activating the FBXW7. (a) The quantification of miR-211-5p by qRT-PCR. (b–e) The abundances of Wnt, *β*-catenin, and cleaved Caspase-3 were quantified by western blot (^∗∗^*P* < 0.01).

**Table 1:** The information of the primers.

Genes	Primers
miR-211-5p-F	5′-ATGCCGCAGCAACATCCAGA-3′
miR-211-5p-R	5′-AGGATGCTGCATGCA CTCGAT-3′
FBXW7-F	5′-ATTGGCAATGAGCGGTTC-3′
FBXW7-R	5′-CGTGGA TGCCACAGGACT-3′
U6-F	5′-CTCGCTTCGGCAGCACA-3′
U6-R	5′-AACGCTTCACGAATTTGCGT-3′

## Data Availability

The datasets used and/or analyzed during the current study are available from the corresponding author on reasonable request.
